The article "Noncoding RNAs and hyperthermic intraperitoneal chemotherapy in advanced gastric cancer" was published in 2022. Journal: Bioengineered.

# Noncoding RNAs and hyperthermic intraperitoneal chemotherapy in advanced gastric cancer

**DOI:** 10.1080/21655979.2021.2021348

**Published:** 2022-01-28

**Authors:** Lisi Zeng, Quanxing Liao, Xiaohui Zeng, Jiacai Ye, Xianzi Yang, Siyu Zhu, Hongsheng Tang, Gaojie Liu, Weiwen Cui, Shaohua Ma, Shuzhong Cui

**Affiliations:** a Institute of Oncology, Affiliated Cancer Hospital & Institute of Guangzhou Medical University, Guangzhou, China; b Department of the Second Area of Gastrointestinal Surgery, Affiliated Cancer Hospital & Institute of Guangzhou Medical University, Guangzhou, China; c Department of Radiotherapy, Affiliated Cancer Hospital and Institute of Guangzhou Medical University, Guangzhou, China; d Department of Medical Oncology, Affiliated Cancer Hospital and Institute of Guangzhou Medical University, Guangzhou, China; e Department of Bioengineering, University of California, Berkeley, California, USA; f Institute of Biopharmaceutical and Health Engineering, Shenzhen International Graduate School, Tsinghua University, Shenzhen, China; g Tsinghua-Berkeley Shenzhen Institute (TBSI), Tsinghua University, Shenzhen, China; h State Key Laboratory of Respiratory Disease, Guangzhou Medical University, Guangzhou, China

**Keywords:** Advanced gastric cancer, hyperthermic intraperitoneal chemotherapy (HIPEC), noncoding RNAs, research progress, prospects

## Abstract

Gastric cancer (GC) is one of the most common malignant tumors globally. About 20–30% of patients with gastric cancer show peritoneal implantation metastasis at the first diagnosis. Peritoneal metastasis is responsible for 70% of deaths of patients with advanced gastric cancer. Although there are many ways to treat advanced gastric cancer, the prognosis of patients with recurrence is unsatisfactory. An auxiliary treatment with hyperthermic intraperitoneal chemotherapy (HIPEC), is an internationally recognized recommended treatment for advanced gastric cancer. A series of clinical trials have shown that HIPEC significantly improves the overall survival of patients with cancer. Compared with the cytoreductive surgery (CRS) alone, HIPEC combined with CRS markedly reduced the rate of peritoneal metastasis in patients with ovarian cancer and colorectal cancer. It has been demonstrated that HIPEC alters transcription of many genes by affecting non-coding RNAs, which may contribute to the suppressive effect of HIPEC on the synthesis of nucleic acids and proteins in cancer cells. This paper reviews the recent advances in understanding the role of non-coding RNAs in tumor invasion and metastasis of advanced gastric cancer. We also consider changes in noncoding RNA levels and other molecules in advanced gastric cancer cases treated with HIPEC. We hope that our review will provide a reference for future research on molecular epidemiology and etiology of advanced gastric cancer and promote precise treatment of this malignancy using HIPEC.

The article "Noncoding RNAs and hyperthermic intraperitoneal chemotherapy in advanced gastric cancer" was published in 2022. Journal: Bioengineered.

## Introduction

According to the latest cancer statistics, gastric cancer is the fifth most common malignancy in the world and the fourth most common cause of cancer-related mortality. Gastric cancer is responsible for over one million new cases in 2020 and an estimated 769,000 deaths[1]. The most important reason for the poor therapeutic effect in patients with gastric cancer is the appearance of peritoneal implantation metastasis [2–4]. Hyperthermic intraperitoneal chemotherapy (HIPEC) is a new adjuvant therapy that significantly reduces the rate of local recurrence and distant metastasis in patients with advanced gastric cancer [5–9]. Noncoding RNAs have become a hotspot in cancer research in recent years. Many studies have shown that noncoding RNAs are closely related to the transmission of drug resistance between tumor cells and tumor microenvironment in a variety of cancers, including advanced gastric cancer. It is therefore necessary to explore changes in noncoding RNA levels following HIPEC as it will provide an important basis for improving HIPEC precision.

Noncoding RNAs play an important role in the occurrence and development of gastric cancer. The therapeutic effect of HIPEC in gastric cancer are associated with noncoding RNAs. Therefore, we reviewed changes in noncoding RNAs in advanced gastric cancer following treatment with HIPEC. We hope our review can provide a reference for future research on molecular epidemiology and etiology of advanced gastric cancer and promote precise treatment of this malignancy using HIPEC.

## Research progress in advanced gastric cancer treatment

Advanced gastric cancer infiltrates into the submucosa, enters the muscular layer, and may pass through the muscular layer to the serosa. After advanced gastric cancer cells infiltrate the muscular layer, or even penetrate into the serosa layer, they can easily spread, resulting in the local dissemination of tumor cells and formation of peritoneal metastasis. Radical surgery is the most commonly used treatment of advanced gastric cancer, which plays an important role in clinical therapy of this disease. At present, the clinical treatment of gastric cancer in our country mainly adopts the comprehensive treatment by using the D2/D3 radical surgery. According to the different objectives and scope of gastric cancer resection, gastric cancer surgery is divided into palliative surgery, extended surgery, and standard radical surgery. In patients with advanced gastric cancer, surgical treatment should aim for complete tumor removal. According to the scope and grouping of peri-gastric lymph node dissection, surgical treatments are classified into D1, D2, and D3 lymph node dissections. D2 lymph node dissection is the standard lymph node dissection recommended by the American Cancer Collaboration Network for the treatment of advanced gastric cancer, and it is the most commonly used lymph node dissection in the clinic. Standard radical gastrectomy accounts for 2% of the total stomach. The indications are N0–N2 (+) with lymph node metastasis, T2–T3 with primary cancer, T1 cancer with diameter larger than 2.0 cm and N1 (+). Standard radical resection can effectively improve the survival rate of patients with advanced gastric cancer without peritoneal metastasis and liver metastasis before and during operation.

The article "Noncoding RNAs and hyperthermic intraperitoneal chemotherapy in advanced gastric cancer" was published in 2022. Journal: Bioengineered.

Because at the early stage, gastric cancer does not manifest clear clinical symptoms, many patients are diagnosed with advanced gastric cancer at the initial diagnosis. About 20–30% of gastric cancer patients present with peritoneal implantation metastasis at the first diagnosis [2]. Importantly, peritoneal implantation metastasis or malignant ascites still predisposes 50% of patients undergoing radical surgery [2,7]. Although great progress has been made in the diagnosis and treatment of gastric cancer in recent years, the prognosis of patients with gastric cancer remains poor. Peritoneal metastasis is the most important cause of death in patients with advanced gastric cancer. Although there are many ways to treat advanced gastric cancer, including surgery, radiotherapy, chemotherapy, biological immunotherapy, and other methods, the prognosis of patients with recurrence is unsatisfactory [3,10–14].

Free cancer cells in the abdominal cavity and postoperative residual microcancer foci are the main factors of peritoneal metastasis of advanced gastric cancer. Free cancer cells reach the intraperitoneal space by several routes. First, when cancer cells from the primary tumor invade the plasma membrane of the gastric wall, they penetrate directly into the abdominal cavity and are planted there or in the adjacent organs. Second, in patients who underwent surgery for advanced gastric cancer, cancer cells from the surgical margin may directly enter the abdominal cavity or get into the severed blood vessels in the operational area. Further, some cancer cells in the lymphatic vessels flow into the abdominal cavity with blood and lymph. Third, the intestinal fluid with exfoliated cancer cells may flow into the abdominal cavity through the cut end of the intestinal loop. In turn, the main sources of the celiac microcancer foci are (1) abdominal microlesions that are invisible to the naked eye and, thus, remaining unresected during the operation, and (2) residual cancer cells that are protected by the fibrin coagulant exuded from the operative field, so that these cells cannot be recognized by immune cells [15].

The article "Noncoding RNAs and hyperthermic intraperitoneal chemotherapy in advanced gastric cancer" was published in 2022. Journal: Bioengineered.

In recent years, several studies pointed out that residual peritoneal cancer cells and microcarcinoma foci found in patients operated for gastric cancer are important causes of recurrence and local metastasis [10]. Finding a way to control peritoneal micrometastasis of advanced gastric cancer is key to successful treatment. Fortunately, hyperthermic intraperitoneal chemotherapy (HIPEC) shows considerable efficacy in this regard and has become an internationally recognized and recommended treatment for advanced gastric cancer [7–9,12,16–18].

## HIPEC reduces recurrence and distant metastasis risk in advanced gastric cancer

HIPEC is an auxiliary procedure in the treatment of peritoneal carcinoma during which a solution containing chemotherapy drugs is infused into the patient’s abdominal cavity at a precise temperature (43°C) and circulated for a certain period of time [19]. HIPEC technology has been continuously improved by researchers and clinical doctors; it evolved from simple perfusion heating and direct infusion to procedures performed at a constant temperature of the perfusate controlled by a water bath. Now HIPEC has become an established technique for precise intraperitoneal heat perfusion after continuous innovation and improvement. HIPEC is typically performed for 60 min at a velocity of perfusion of 450–600 mL/min and an inflow temperature of 43 ± 0.2°C [6,20,21]. High-precision, high-volume, and continuous circulation therapies have been established on the basis of HIPEC. This technique is used to remove free peritoneal cancer cells, subclinical lesions, and microcancer nodules, offering hope to patients with advanced gastric cancer who have peritoneal metastasis.

Precision HIPEC is based on three principles. First, accurate temperature control is essential: available *in vitro* and *in vivo* double circulation temperature control technology achieves temperature control accuracy within ±0.1°C, with flow rate control variation within ±5%. Second, accurate treatment location is achieved by placing four perfusion tubes under the diaphragm and pelvic floor of the abdominal cavity through the para-colonic groove, so that the hot perfusion fluid fills the whole abdominal cavity, leaving no unperfused areas and maximizing the therapeutic effect of HIPEC. Third, accurate clearance ensures that warm perfusion fluid at a constant temperature accurately removes free cancer cells, subclinical lesions, and microcancerous nodules of less than 40 μm, so that they can no longer enter the abdominal cavity of patients after clearance and filtration. The synergistic effect of heat and chemotherapy kills free cancer cells in the abdominal cavity [16]. Some clinical trials also confirmed that peritoneal lavage cytology became negative after HIPEC [22].

The article "Noncoding RNAs and hyperthermic intraperitoneal chemotherapy in advanced gastric cancer" was published in 2022. Journal: Bioengineered.

HIPEC mainly uses the dual effects of hyperthermia and chemotherapy to treat cancer. Intraperitoneal chemotherapy results in a high concentration of cytotoxic drugs in the abdominal cavity. Hyperthermia likely enhances the effects of intraperitoneal chemotherapy in two ways: (1) by increasing the sensitivity of tumor cells to chemotherapy drugs and (2) by exerting direct cytotoxic effects, such as the damage of DNA repair mechanisms, denaturation of proteins, inhibition of oxidative mechanism, and increased lysosomal activity [5,16]. Therefore, HIPEC plays an important role in inhibiting postoperative recurrence and metastasis of advanced gastric cancer. The principles of drug selection for HIPEC should consider not only the types of the primary disease, but also the sensitivity of patients. The characteristics of the drugs, such as drug penetration into abdominal tumors, peritoneal absorption should also be taken into account. Various drugs have been used for HIPEC, including paclitaxel, docetaxel, oxaliplatin, cisplatin, 5-fluorouracil, and epirubicin [23–25].

A clinical study of patients with advanced gastric cancer at the Ruijin Hospital in Shanghai showed that HIPEC reduced the incidence of peritoneal recurrence of this malignancy by 24%, improving the median survival by 18 months [26]. Through a retrospective study, Zhang et al. demonstrated that HIPEC was superior to intravenous chemotherapy alone in controlling postoperative recurrence and metastasis of advanced gastric cancer. In that study, in 3 years after the operation, the peritoneal metastasis rate in the HIPEC group was 16.2%, which was significantly lower than 38.5% in the intravenous chemotherapy group [27]. A systematic review of published reports indicated that a combination of cytoreductive surgery (CRS) and HIPEC can improve prognosis in patients with advanced gastric cancer [28]. In summary, HIPEC has advantages in the clinical treatment of peritoneal metastasis of advanced gastric cancer.

Continuous breakthroughs have been made in developing the theoretical basis behind HIPEC and in its technical execution. In 2014, the International Conference on Peritoneal Cancer in Amsterdam (the Netherlands) adopted CRS combined with HIPEC as the standard treatment for mucinous carcinoma of the appendix, peritoneal metastasis of colorectal cancer, and malignant mesothelioma, and as a recommended treatment for ovarian cancer and gastric cancer with peritoneal metastasis [29]. After the first multicentre randomized controlled clinical trial of HIPEC for the treatment of advanced ovarian cancer was reported in New England Journal of Medicine in 2018, the FIGO Cancer report in 2018 included HIPEC in the guidelines for the diagnosis and treatment of ovarian cancer. The first edition of NCCN in 2019 also included HIPEC in the guidelines for the treatment of ovarian cancer. The American Anti-Cancer Association also recommends HIPEC as a treatment for patients with peritoneal metastasis of gastric cancer [30].

The article "Noncoding RNAs and hyperthermic intraperitoneal chemotherapy in advanced gastric cancer" was published in 2022. Journal: Bioengineered.

## Noncoding RNAs in gastric cancer

It has been well established that gastric cancer has genetic and environmental causes. Early conventional molecular epidemiology studies reported that precancerous lesions, tumor formation, and invasion and metastasis of gastric cancer were associated with environmental risk factors. A study from the National Cancer Institute found a significant positive correlation between the risk of non-cardiac gastric cancer and serum gastrin levels [31]. Recently, clinical data showed that some substances in blood have been linked to the development of gastric cancer, such as pepsinogen, *Helicobacter pylori*, growth hormone releasing peptide. Because they contribute to the development of gastric cancer, they may be used as serum or plasma markers for the early detection of gastric cancer [32–34]. Traditional screening for gastric cancer markers such as CA19-9, CEA, and CA72-4, detects nonspecific tumor-associated antigens with low specificity and low diagnostic rate [35].

Nowadays, with the development of molecular detection technologies, a greater number of biomarkers associated with gastric cancer can be detected. Studies of non-coding RNA and protein markers based on microarrays have indicated that microRNAs (miRNAs), long non-coding RNAs (lncRNAs), and circular RNAs (circRNAs) play an important role in various biological processes, such as proliferation, differentiation, apoptosis, and migration of tumor cells. By direct or indirect regulation of DNA transcription, they act as regulators of growth and development of living organisms [36–38].

Noncoding RNAs mainly include miRNAs, lncRNAs, and circRNAs [39–41]. Competing endogenous RNA (ceRNA) hypothesis links the function of noncoding RNAs with that of protein-coding mRNAs. CeRNA hypothesis proposes that protein-coding mRNAs, miRNAs, lncRNAs, and circRNAs can function as miRNA sponges via their multiple miRNA binding sites [42,43]. With high tumor relevance, tissue specificity, and expression in blood cells, miRNAs, lncRNAs, and circRNAs may be an ideal method for detection of tumor material in blood. Li et al. found that miR-199a-3p is one of the best tumor markers, with an accuracy of 75% and a sensitivity of 76% in the diagnosis of early gastric cancer [44]. Kim et al. confirmed that *miR-1* and *miR-34* were closely related to drug resistance of gastric cancer cells, so their levels can used for the evaluation of drug resistance and chemotherapeutic sensitivity in patients with gastric cancer [45]. Fattahi et al. found that the expression of *LINC00152* was significantly higher in gastric cancer cells than that of normal gastric cells. Because the level of *LINC00152* has high sensitivity and specificity in the diagnosis of gastric cancer, it may be used as a tumor marker [38]. Further research conducted by Zhao et al. found that knockdown of *LINC00152* inhibited cell migration and invasion [46]. The research by Xie et al. showed that *ciRS-7*, a novel circRNA, inhibited the invasion of tumor cells by blocking the function of miR-7 [47]. There are also other noncoding RNAs relevant for gastric cancer manifestations (Figure 1; Table 1).

The article "Noncoding RNAs and hyperthermic intraperitoneal chemotherapy in advanced gastric cancer" was published in 2022. Journal: Bioengineered.

**Table 1.** Related noncoding RNAs in gastric cancer of this review

Type of ncRNAs	Expression	Putative roles	Pathway	Targets	Ref
**lncRNAs**					
LINC00152	Upregulated	Promote proliferation and colony formation	EMT	E-cadherin	[39]
HOTAIR	Upregulated	Lmphatic metastasis	H3K27 methylation	H3K27	[53]
DKFZP434K028, RPL34-AS1	Downregulated	Potential biomarker	Unknown	MYRF	[47]
LINC01133	Downregulated	EMT/ metastasis	Wnt/β-catenin	miR-106a-3p/ APC	[54]
XLOC_006753	Upregulated	Promote drug resistance	mTOR/PI3K/AKT signaling	Unknown	[55]
lncR-D63785	Downregulated	Promote drug resistance	mTOR/PI3K/AKT signaling	miR-422/MEF2D	[56]
ZFAS1	Upregulated	Promote proliferation and migration	EMT	KLF2 and NKD2	[57]
Lnc-GNAQ-6:1	Downregulated	Potential biomarker	Unknown	Unknown	[58]
lncSLC2A12-10:1	Upregulated	Potential biomarker	Unknown	Unknown	[59]
LINC00483	Upregulated	Promote invasion and migration	Unknown	miR-490-3p/MAPK1	[60]
lncRNA HCP5	Upregulated	Promote proliferation, invasion, and migration	Unknown	miR-299-3p/SMAD5	[62]
LINC00240	Upregulated	Promote proliferation and migration	Unknown	miR-338-5p/METTL3	[63]
LINC01320	Upregulated	Promote aggressive phenotype	Unknown	miR-495-5p/RAB19	[64]
CERS6-AS1	Upregulated	Promote proliferation, migration and invasion	Unknown	Unknown	[65]
LINC00511	Upregulated	Promote proliferation and migration	Unknown	microRNA-625-5p/STAT3	[66]
PCED1B-AS1	Upregulated	Promote proliferation, migration, invasion and EMT	Unknown	microRNA-215-3p/C-X-C motif chemokine receptor 1	[67]
LINC00649	Upregulated	Promote proliferation, migration and EMT	YAP1/Hippo pathway	miR-16-5p	[68]
NR2F1-AS1	Upregulated	Promote proliferation, invasion and migration	Unknown	SPI1/ST8SIA1	[69]
AL139002.1	Upregulated	Promote proliferation, migration, invasion, and EMT	Unknown	microRNA-490-3p Hepatitis A Virus Cellular Receptor 1	[70]
LINC00265	Upregulated	Promote proliferation	Unknown	microRNA-144-3p/Chromobox 4	[71]
MYLK-AS1	Upregulated	Promote proliferation, migration, and invasion	Unknown	LATS2	[72]
BC031243	Upregulated	CRS + HIPEC	Unknown	Unknown	[107]
RP11-356I2.2	Upregulated	CRS + HIPEC	Unknown	Unknown	[107]
**miRNAs**					
miR-199a-3p	Upregulated	Promote invasion and migration	Unknown	ETNK1, ZHX1	[45]
miR-1, miR-34	Downregulated	Inhibit drug resistance	Unknown	Sorcin	[46]
miR-100-3p	Downregulated	Inhibit proliferation and apoptosis	Bax/Bcl2/Caspase3	BMPR2	[75]
miR-221	Upregulated	lymph node metastasis	p-JAK2, p-STAT3	SOCS3	[76]
miR-423-5p	Upregulated	lymph node metastasis	Unknown	SUFU	[77]
miR-3189-3p	Downregulated	CRS + HIPEC	Unknown	CFL2	[106]
miR-1825	Downregulated	CRS + HIPEC	Unknown	Unknown	[106]
miR-32-3p, miR-3149, miR-4297	Upregulated	CRS + HIPEC	Unknown	Unknown	[106]
miR-1299	Upregulated	CRS + HIPEC	Unknown	ETS1	[106]
miR-218	Upregulated	CRS + HIPEC	SMO signaling	Gli2	[107]
miR-8-3p	Upregulated	HIPEC	AMPK signaling	PPP2R5B	[110]
miR-23a	Downregulated	Heat-stressed	Unknown	NOXA	[112]
miR-10b	Downregulated	Hyperthermia	Unknown	Hoxd10	[113]
miR-15b	Downregulated	Hyperthermia	DYNLT1/Caspase-3/Caspase-9 signaling	DYNLT1	[113]
miR-106a	Upregulated	Promote growth	Unknown	Smad7	[78]
miR-425	Upregulated	Promote cell viability, migration, and invasion	Unknown	Dickkopf-related protein-3	[79]
miR −1269b	Downregulated	Inhibit proliferation, migration, and invasion	Unknown	METTL3	[80]
miR-130a-3p	Upregulated	Promote proliferation, migration, and invasion	Unknown	GCNT4/TGF-beta1/SMAD3	[81]
**circRNAs**					
ciRS-7	Upregulated	Inhibit the invasion	PTEN/PI3K/AKT Signaling	miR-7	[48]
circ-PVT1	Upregulated	Promote drug resistance	Unknown	miR-124/ZEB1	[84]
circ-MTHFD2	Upregulated	Promote drug resistance	Unknown	miR-124	[85]
circ-OXCT1	Downregulated	Suppress EMT progress	Unknown	miR-136/SMAD4	[86]
circCCDC9	Downregulated	Inhibit the proliferation, migration and invasion	Unknown	miR-6792-3p/CAV1	[87]
circ-RanGAP1	Upregulated	promotes GC progression	Unknown	miR-877-3p/VEGFA	[88]
circSHKBP1	Upregulated	Promote proliferation, invasion and migration	miR-582-3p/HUR/VEGF	miR-582-3p	[89]
circRNA_102231	Upregulated	Promote proliferation and invasion	Unknown	IRTKS	[90]
hsa_circ_0000751	Downregulated	Inhibit progression, migration, and invasion	Unknown	miR-488/UQCRC2	[91]
circPRKDC	Upregulated	Promote cell viability, metastasis, and EMT	Unknown	IRS2/microRNA-493-5p	[92]
circ-HN1	Upregulated	Promote proliferation, migration, and invasion	miR-485-5p/GSK3A pathway	Unknown	[93]
hsa_circ_0000117	Upregulated	Promote proliferation and invasion	Unknown	microRNA-337-3p/signal transducer and activator of transcription 3 axis	[94]
circCOL6A3_030	Upregulated	Promote migration	Unknown	Unknown	[95]
circ0005654	Upregulated	Promote proliferation, migration and invasion	Unknown	miR-363/sp1/myc/Wnt/β-catenin axis	[96]

The article "Noncoding RNAs and hyperthermic intraperitoneal chemotherapy in advanced gastric cancer" was published in 2022. Journal: Bioengineered.

**Figure 1.** Noncoding RNAs relevant to cell gene functions in gastric cancer.

## LncRNAs in advanced gastric cancer

LncRNAs are a group of RNA polymerase II transcripts with a length of >200 nucleotides. Most of lncRNAs lack obvious open reading frames and therefore, do not encode proteins. Recently, it has been demonstrated that some lncRNAs can encode stable, functional small peptides (also known as micropeptides) [48]. According to the position of the chromosome, lncRNAs can be divided into five types: sense, antisense, intergenic, bi-directional, and intragenic lncRNAs. In recent years, a large number of studies have shown that lncRNA plays an important regulatory role in tumor biological characteristics through the transcriptional and post-transcriptional mechanisms [49,50]. LncRNA modifies chemoresistance by regulating different target genes. For example, lncRNA *PCAT-1* is overexpressed in cisplatin-resistant gastric cancer tissues and cells, where it promotes resistance to cisplatin by affecting the *miR-128*/ZEB1 axis [51]. LncRNA *HOTAIR* promotes resistance of gastric cancer cells to adriamycin via inhibition of *miR-217* expression [52]. It has been shown that reduced expression of lncRNA *LINC01133* is associated with aggressive tumor phenotypes and poor patient outcomes in gastric cancer, because *LINC01133* inhibits gastric cancer progression and metastasis by acting as a ceRNA for *miR-106a-3p* to regulate APC expression and the Wnt/β-catenin pathway [53]. Zeng et al. have demonstrated that high expression of *XLOC_006753* promoted the development of multi-drug resistance (MDR) via activation of the PI3K/AKT/mTOR pathway in gastric cancer cells [54]. Wang et al. have shown that lncRNA *CRAL* was downregulated in cisplatin-resistant GC cells, which attenuated the extent of cisplatin-induced DNA damage and cell apoptosis and thus contributed to cisplatin resistance in GC cells [55]. It emerged that *CRAL* could function as a ceRNA for endogenous *miR-505*, thereby upregulating expression of cylindromatosis (CYLD), which, in turn, suppressed AKT activation and enhanced the sensitivity of gastric cancer cells to cisplatin via the miR-505/CYLD/AKT axis. These observations suggested that *CRAL* could be considered a potential predictive biomarker and therapeutic target for cisplatin resistance in gastric cancer [55]. Pan et al. demonstrated high expression of lncRNA *ZFAS1* in highly metastatic gastric cancer cells and showed that there was increased level of lncRNA *ZFAS1* in tumor tissues, serum, and serum exosomes. The increased expression of *ZFAS1* significantly correlated with lymphatic metastasis and TNM stage. *ZFAS1* knockdown inhibited cell cycle progression, induced apoptosis, and suppressed epithelial-interstitial transformation EMT, which overall attenuated the proliferation and migration of gastric cancer cells [56]. On the contrary, overexpression of *ZFAS1* promoted the proliferation and migration of gastric cancer cells [56]. LncRNA *GNAQ-6:1*, which inhibited apoptosis and promotes cell proliferation, migration, and invasion of gastric cancer cells may also be a potential biomarker in the diagnosis and prognosis of gastric cancer [57]. Zheng et al. found that exosomal lncRNA *SLC2A12-10:1* was a diagnostic biomarker for gastric cancer, and its level predicted patient prognosis [58]. Luo et al. showed that lncRNA *LINC00483* affected the migration and invasion ability of gastric carcinoma cells likely by acting as a ceRNA that competitively sponged *miR-490-3p* to regulate MAPK1 expression [59]. Zhou et al. found that downregulation of lncRNA D63785 suppressed proliferation, migration, and invasion capacities of gastric carcinoma cells [60]. Yin et al. found that downregulation of lncRNA *HCP5* inhibited gastric cancer cell proliferation, invasion, and migration via regulation of the *miR-299-3p*/*SMAD5* axis [61]. Wang et al. demonstrated that *LINC00240* was highly expressed in gastric cancer tissues and cells, and its knockdown inhibited gastric cancer cell proliferation and migration by modulating the *miR-338-5p*/*METTL3* axis [62]. Hu et al. showed that *LINC01320* overexpression promote the aggressive phenotype of gastric cancer cells via the regulation of the *miR-495-5p*/*RAB19* axis [63]. Other studies have also shown that lncRNAs *CERS6-AS1, LINC00511, PCED1B-AS1, LINC00649, NR2F1-AS1, AL139002.1, LINC00265*, and *MYLK-AS1* might promote the progression of gastric cancer and therefore, have the potential to be novel therapeutic targets for treating gastric cancer [64–71].

The article "Noncoding RNAs and hyperthermic intraperitoneal chemotherapy in advanced gastric cancer" was published in 2022. Journal: Bioengineered.

## MiRNAs in advanced gastric cancer

MiRNAs are a class of single-stranded non-coding RNA molecules with a length of about 20 to 24 nucleotides that regulate gene expression by inhibiting mRNA stability and interfering with translation. It has been shown that miRNAs play an important role in the occurrence and development of gastric cancer. Treatments for gastric cancer mainly include surgery, radiation therapy, and chemotherapy. Surgery is the primary treatment for patients at an early stage of gastric cancer, whereas chemotherapy is the main treatment for advanced disease. However, chemotherapy resistance frequently occurs in patients with advanced gastric cancer. This restricts the clinical benefit of the chemotherapeutic agents, and it is one of the main reasons for the failure of gastric cancer treatment [10,72,73]. The mechanisms of drug resistance in gastric cancer are being increasingly better understood, and miRNAs are thought to play a very important role in this process. It was found that production of exosomes in gastric cancer cells was significantly higher than that in normal gastric epithelial cells, and the expression levels of *miR-100* and *miR-148* in exosomes of gastric cancer cells were higher than those in normal gastric epithelial cells [74]. Wang et al. found that *miR-214, miR-221*, and *miR-222* in gastric cancer cells are usually upregulated in gastric cancer tissue-derived mesenchymal stem cells (GC-MSCs) and tissues. Their levels are closely related to lymph node metastasis, venous invasion, and TNM stage. MSCs derived from gastric cancer tissue significantly promoted the growth and migration of HGC-27 human gastric carcinoma cells and increased *miR-221* levels by paracrine secretion. Furthermore, GC-MSC-specific disruption of *miR-221* blocked the tumor-supporting effect of these cells. It was found that GC-MSC-derived exosomes could transfer *miR-221* to HGC-27 cells and promote their proliferation and migration [75]. Li et al found that serum level of *miR-423-5p* in patients with gastric cancer was increased and significantly correlated with lymph node metastasis. High level of *miR-423-5p* is associated with poor prognosis in patients with gastric cancer. *MiR-423-5p* can be internalized into gastric cancer cells, which was shown to enhance their proliferation and migration capacities. Further mechanistic studies showed that *miR-423-5p* inhibited the expression of suppressor of fusion protein (SUFU) and thereby augmented proliferation and migration of gastric cancer cells [76]. Zhu et al. found that exosomal *miR-106a* interacts with Smad7, affects the structure and function of peritoneal mesothelial cells, and promotes peritoneal metastasis [77]. Pei et al. showed that *miR-425* is highly expressed in gastric cancer and that its downregulation suppressed viability, migration, and invasion properties of cancer cells [78]. Kang et al. found that *miR-1269b* overexpression inhibited proliferation, migration, and invasion of gastric cancer cells [79], whereas Hu et al. demonstrated that overexpression of *miR-130a-3p* facilitated these tumourigenic processes [80].

The article "Noncoding RNAs and hyperthermic intraperitoneal chemotherapy in advanced gastric cancer" was published in 2022. Journal: Bioengineered.

## CircRNAs in advanced gastric cancer

CircRNAs are covalently closed non-coding RNAs that regulate gene expression in eukaryotes. High-throughput RNA sequencing and bioinformatics methods have revealed that there is a large number of circRNAs in human cells. Many circRNAs have certain tissue and timing specificity and are closely related to physiological development and various diseases, such as cancer [81]. CircRNA has been proved to be enriched and stable in the cytoplasm, indicating its potential as a tumor biomarker. In contrast to the linear RNA, circRNA has a covalently closed ring structure formed by trans-splicing, which makes it highly stable and biologically conservative. Recent studies have shown that circRNAs are abnormally expressed in a variety of tumor tissues, where they regulate cancer cell proliferation, invasion, and apoptosis, acting as miRNA sponges. Therefore, circRNA may become a new diagnostic marker and a potential therapeutic target [82]. Recent studies have found that circRNAs indirectly affect the occurrence and development of gastric cancer. Liu et al. found that circRNA *circ-PVT1* was upregulated in gastric cancer cells, and this upregulation could cause their increased resistance to paclitaxel, as *circ-PVT1* sponged *miR-124-3p*, which led to increased expression of zinc finger E-box binding homeobox 1 [83]. In addition, knockdown of *circ-PVT1* enhanced the sensitivity of paclitaxel-resistant gastric cancer cells to paclitaxel. Xu et al. showed that direct binding of *circ-MTHFD2* to *miR-124* through the molecular sponge effect increased the expression of the MDR-1 protein and enhanced drug resistance of MGC-803/MTA cells [84]. Liu et al. found that *circ-OXCT1* overexpression inhibited gastric cancer EMT progress by competitively sponging *miR-136*, which implied that manipulating *circ-OXCT1* levels could be a novel treatment for advanced gastric cancer [85]. Luo et al. showed that upregulation of *circ-CCDC9* suppressed proliferation, migration, and invasion abilities of gastric carcinoma cells. *Circ-CCDC9* could be a potential biomarker for patients with gastric cancer [86]. Lu et al showed that *circ-RanGAP1* promoted gastric cancer progression by competitively sponging *miR-877-3p*, whereas the downregulation of *circ-RanGAP1* inhibited tumor growth and metastasis of gastric cancer [87]. Xie et al. found that exosomal *circ-SHKBP1* suppressed HSP90 degradation and promoted gastric cancer progression by regulating the *miR-582-3p*/HUR/VEGF pathway [88]. Yuan et al. showed that *circRNA_102231* silencing inhibited gastric cancer cell proliferation and invasion and that this circRNA could also act as a potential biomarker and therapeutic target in gastric cancer patients [89]. Wang et al. demonstrated that *hsa_circ_0000751* was downregulated in gastric cancer tissues and cell lines, whereas *hsa_circ_0000751* overexpression suppressed tumor progression as well as migration and invasion capacities of cancer cells [90]. Other circRNAs, such as *circPRKDC, circ-HN1, hsa_circ_0000117, circCOL6A3*_*030*, and *circ0005654* have been suggested to accelerate gastric cancer development, so they might also become novel potential targets for gastric cancer treatment [91–95].

The article "Noncoding RNAs and hyperthermic intraperitoneal chemotherapy in advanced gastric cancer" was published in 2022. Journal: Bioengineered.

CircRNAs participate in a variety of metabolic and signal transduction pathways closely related to drug resistance in gastric cancer, and can specifically regulate the expression of tumor-related genes. These studies not only have improved our understanding of the molecular characteristics of gastric cancer, but also provided new ideas for molecular targeted therapy of gastric cancer aimed at circRNAs.

## Noncoding RNAs are involved in many signaling pathways in gastric cancer

Among the oncogenic pathways involved in the emergence and development of gastric cancer are the PI3K/AKT/mTOR, Wnt/β-catenin, NF-κB, MAPK, Notch, and inflammatory signaling pathways (Figure 2), which could be regulated by noncoding RNAs. The PI3K/AKT/mTOR signaling is one of the most frequently dysregulated pathways in gastric cancer. Previous studies have revealed that noncoding RNAs play an important role in regulating the PI3K/AKT/mTOR signaling pathway through targeting its key molecules. Chen et al. showed that the activation of the phosphoinositide 3-kinase, serine/threonine kinase Akt, mammalian target of rapamycin (PI3K/Akt/mTOR), and mitogen-activated protein kinase (MAPK) pathways might be the reason for above phenotypic alternations [96]. Lu et al provided a new insight that CD133 activates the PI3K/AKT/mTOR signaling transduction pathway, resulting in the inhibition of autophagy and increased cisplatin resistance of Cis-KATO-III cells [97]. Tian et al. demonstrated that *miR-361-5p* suppressed autophagy-induced chemoresistance of gastric cancer cells through targeting FOXM1 via the PI3K/Akt/mTOR pathway, providing a potential novel avenue for treatment of gastric cancer [98]. Cheng et al. showed that *HOTAIR* knockdown inhibited cisplatin resistance of gastric cancer cells by upregulating *miR-34a* through the PI3K/Akt and Wnt/β-catenin signaling pathways [99]. Liu et al. found that inhibition of the Wnt/β-catenin pathway by ICG-001, a specific Wnt/β-catenin inhibitor, preferentially reduced proliferation and invasion of trastuzumab-resistant cells and reversed EMT [100]. Thus, given that the Wnt/β-catenin pathway mediates trastuzumab resistance, the combination of Wnt/β-catenin inhibitors with trastuzumab may be an effective treatment option [100]. Yang et al. demonstrated that *BATF2* was downregulated in MDR gastric cancer cells, whereas *BATF2* overexpression reversed the MDR of gastric cancer cells by inactivating the Wnt/β-catenin pathway [101]. Fu et al. showed that downregulation of the NIBP protein by *Ginkgo biloba* extract 761 suppressed the cis‑diamminedichloroplatinum (II)‑induced activation of the NF‑κB signaling pathway, EMT, and CD133 expression [102]. Zhuang et al showed that conditioned medium (cm) from cultures of SGC‑7901 gastric carcinoma cells activated the ataxia‑telangiectasia mutated (ATM) and NF‑κB pathways and upregulated expression levels of ATP‑binding cassette subfamily G member 2 and MDR‑associated protein 2, thereby augmenting chemotherapeutic resistance of SGC‑7901cells [103]. Wang et al found that 25‑hydroxycholesterol, an oxysterol derivative of cholesterol involved in inflammation, immune responses, and cancer development, promoted invasion of gastric cancer cells by upregulating TLR2/NF‑κB‑mediated matrix metalloproteinase expression [104]. The molecular mechanism of tumor drug resistance is very complex and includes abnormal expression of transporter super family proteins, inhibition of apoptosis, abnormal activation of signaling pathways, and other factors. Signal transduction pathways affect tumor formation, development, metastasis, and invasiveness. A full understanding of signaling pathways mediating tumor drug resistance in gastric cancer can help develop novel therapeutics that would restore drug sensitivity of tumor cells with high efficiency, high selectivity, and low risk of adverse reactions.

The article "Noncoding RNAs and hyperthermic intraperitoneal chemotherapy in advanced gastric cancer" was published in 2022. Journal: Bioengineered.

**Figure 2.** Involvement of noncoding RNAs in the classical signaling pathways, such as PI3K/AKT/mTOR, Wnt/β-catenin, NF-κB, MAPK, and Notch, and in the inflammatory signaling pathways in gastric cancer.

## Noncoding RNAs and HIPEC in advanced gastric cancer

HIPEC mainly kills tumor cells by continuous mechanical scouring and improving immunity through hyperthermia, chemotherapy, and the synergistic effect of both. HIPEC thermal effects include not only enhanced sensitivity of tumor cells to chemotherapeutic drugs, but also suppressed angiogenesis in cancer tissue as well as activation of tumor cell degeneration and necrosis. At the molecular level, HIPEC denatures cancer cell membrane proteins and interferes with DNA, RNA, and protein synthesis (Figure 3) [105]. Abnormally expressed noncoding RNAs can also be a factor in HIPEC therapy [15]. Zeng et al. showed that lncRNAs were differentially expressed following the treatment with CRS + HIPEC, suggesting that they might play key roles in tumor development. A high-throughput microarray analysis was performed to compare expression profiles of lncRNAs and mRNAs in advanced gastric cancer serum samples after CRS + HIPEC. PCR results further verified that eight lncRNAs were aberrantly expressed in advanced gastric cancer serum samples after CRS + HIPEC compared with the matched serum sample before CRS + HIPEC [106]. Zhang et al. found that *miR-218* was upregulated in gastric cancer after HIPEC, which was associated with increased chemosensitivity to cisplatin. Hierarchical clustering of microRNAs in advanced gastric cancer serum samples showed that *miR-218, miR-3189-3p, miR-1825, miR-2115-5p* and several other microRNAs were upregulated after HIPEC, whereas *miR-32-3p, miR-3149, miR-4297, miR-1299* and several other microRNAs were downregulated. Zeng et al. reported that lncRNAs were differentially expressed after CRS + HIPEC, suggesting that they might play key roles in tumor development. Their results also indicated that targeting *miR-218* may provide a strategy for blocking the development of gastric cancer in conjunction with HIPEC treatment [107]. Ruan et al. demonstrated that thermo-chemotherapy effectively decreased the invasion capability of cancer cells, increased cell-cell adhesion and E-cadherin expression, as well as upregulated *miR-218* expression, which correspondingly decreased the expression of the *miR-218* downstream target Gli2. Their results further clarified the possible role of *miR-218* in HIPEC [108], implying that HIPEC effects on tumor cells include changes in the expression of noncoding RNAs. Feng et al. found that precise hyperthermia upregulated *miR-409-3p* and KLF17, which promoted apoptosis and inhibited migration, invasion, and EMT of gastric cancer cells [109]. Thus, HIPEC can affect tumor cells by regulating the expression of microRNAs [109].

**Figure 3.** Changes in the levels of noncoding RNAs and cell functions in gastric cancer after treatment with HIPEC.

The thermal effect, similar to that of HIPEC, can also be seen in other similar heat treatment experiments. Hu et al. showed that hyperthermia (43°C for 30 min) promoted lactate secretion by inhibiting phosphorylation of adenosine monophosphate-activated protein kinase (AMPK) in cultured immature boar Sertoli cells. *miR-8-3p* was shown to act as a novel regulator of AMPK-modulated lactate secretion by targeting PPP2R5B in hyperthermic boar Sertoli cells [110]. Zhang et al. found that high temperature over the thermoneutral zone of sows during the summer increased the serum level of heat shock protein 70 (HSP70) and decreased the activity of superoxide dismutase. In this study, by using RNA sequencing and bioinformatics analysis, it was shown that 59 circRNAs were differentially expressed as a result of high temperature, including 42 upregulated and 17 downregulated circRNAs in pituitaries of the heat-stressed sows [111]. Roufayel et al. demonstrated that *miR-23a* levels decreased in heat-stressed cells, which correlated with an increased abundance of *NOXA* mRNA, whereas the elimination of *miR-23a* in heat-stressed cells could be prevented by HSP70 [112]. Erves et al. found that hyperthermia-dependent attenuating influence on three distinct breast cancer-related microRNAs *in vitro* had translational potential for clinical breast cancer treatment, because the identified microRNAs *miR-10b, miR-15b*, and *miR-139* are known to have oncogenic as well as tumor suppressor functions in breast cancer [113].

The article "Noncoding RNAs and hyperthermic intraperitoneal chemotherapy in advanced gastric cancer" was published in 2022. Journal: Bioengineered.

However, the mechanism whereby noncoding RNAs, including lncRNAs, miRNAs, and circular RNAs, can be utilized in the treatment of advanced gastric cancer and other cancer cells by HIPEC remains to be further explored.

## Discussion

As a new adjuvant therapy, HIPEC can significantly reduce the rate of local recurrence and distant metastasis in patients with advanced gastric cancer. HIPEC provides an effective treatment for peritoneal implantation metastasis that cannot be fully treated by surgery and, thus, has become an indispensable technology in the field of gastric cancer treatment. Combination of HIPEC with surgical treatment provides a scientifically justified and reasonable way of gastric cancer treatment. At present, however, domestic and foreign experts have insufficient understanding of the technical advantages and mechanism(s) of action of HIPEC, although many medical centers at home and abroad are carrying out clinical studies on the prevention of peritoneal cancer by utilizing this technique. However, for proper evidence-based medicine, multicentre randomized controlled clinical trials are still needed to confirm the role and significance of HIPEC in the prevention and treatment of advanced gastric and peritoneal cancer. HIPEC also needs to be more accurate and its optimization can be achieved with the help of molecular biology approaches.

## Conclusions

An increasing number of noncoding RNAs has been shown to be involved in the development of gastric cancer. In order to achieve curation by using HIPEC in the clinical setting, a risk prediction model for the progression and prognosis of advanced gastric cancer should be established through a comprehensive evaluation of molecular changes relevant to this malignancy, among which non-coding RNAs likely play an important role. Treatments targeting noncoding RNAs abnormally expressed in gastric cancer may be a promising approach to augment the efficacy of HIPEC.

The article "Noncoding RNAs and hyperthermic intraperitoneal chemotherapy in advanced gastric cancer" was published in 2022. Journal: Bioengineered.

## Highlights

Recent progress in advanced gastric cancer treatment is discussed.

HIPEC reduces recurrence and distant metastasis risk in advanced gastric cancer.

Abnormally expressed ncRNAs are involved in gastric cancer and HIPEC efficacy.
